# Medical Internet of Things to Realize Elderly Stroke Prevention and Nursing Management

**DOI:** 10.1155/2021/9989602

**Published:** 2021-07-06

**Authors:** Xin Li, Sufen Ren, Fangqiu Gu

**Affiliations:** School of Nursing Jinzhou Medical University, Jinzhou, Liaoning 121000, China

## Abstract

Stroke is a major disease that seriously endangers the lives and health of middle-aged and elderly people in our country, but its implementation of secondary prevention needs to be improved urgently. The application of IoT technology in home health monitoring and telemedicine, as well as the popularization of cloud computing, contributes to the early identification of ischemic stroke and provides intelligent, humanized, and preventive medical and health services for patients at high risk of stroke. This article clarifies the networking structure and networking objects of the rehabilitation system Internet of Things, clarifies the functions of each part, and establishes an overall system architecture based on smart medical care; the design and optimization of the mechanical part of the stroke rehabilitation robot are carried out, as well as kinematics and dynamic analysis. According to the functions of different types of stroke rehabilitation robots, strategies are given for the use of lower limb rehabilitation robots; standardized codes are used to identify system objects, and RFID technology is used to automatically identify users and devices. Combined with the use of the Internet and GSM mobile communication network, construct a network database of system networking objects and, on this basis, establish information management software based on a smart medical rehabilitation system that takes care of both doctors and patients to realize the system's Internet of Things architecture. In addition, this article also gives the recovery strategy generation in the system with the design method of resource scheduling method and the theoretical algorithm of rehabilitation strategy generation is given and verified. This research summarizes the application background, advantages, and past practice of the Internet of Things in stroke medical care, develops and applies a medical collaborative cloud computing system for systematic intervention of stroke, and realizes the module functions such as information sharing, regional monitoring, and collaborative consultation within the base.

## 1. Introduction

Stroke is a sudden onset of cerebral blood circulation disorders. It is divided into ischemic stroke and hemorrhagic stroke. Among them, ischemic stroke accounts for about all strokes—80% [1]. Stroke is a major disease that seriously endangers the lives and health of middle-aged and elderly people in our country. Its incidence, recurrence, disability, and fatality rate are extremely high. It not only endangers the lives of patients, but also brings heavy burdens to the patients' families and society economic burden [2]. The National Health and Family Planning Commission's Stroke Screening and Prevention Engineering Committee has carried out a nationwide stroke high-risk screening project to identify high-risk groups. The follow-up work is to further prevent strokes for high-risk groups. The focus should be on early stroke patients. Discovery, early diagnosis, and early treatment (secondary prevention) are on [3]. However, domestic and foreign surveys have shown that the rate of timely medical treatment for stroke is very low, and the implementation of secondary prevention needs to be improved [4]. Ischemic stroke is the most common type of stroke, accounting for 60% to 80% of strokes [5]. The results of domestic studies show that the incidence of ischemic stroke is 91.3 to 263.1 per 100,000, the average annual incidence is 14.55 per 100,000, and the recurrence rate is 8.47% [6]. A 6-year follow-up study showed that the fatality rate for the first stroke was 74.3% (919/1 237), and the average annual fatality rate was 12.3% [7]. The high incidence of stroke, high recurrence rate, high disability rate, and high fatality rate seriously threaten human health, and it has also become the focus of medical workers' attention [8]. Stroke is preventable, controllable, and treatable, but the span from primary prevention to acute treatment to secondary prevention is relatively large, and the actual clinical management and control is time-consuming, laborious, and inefficient. The development of information technology provides a new opportunity to manage stroke patients across time and space [9]. At present, there have been studies on the application of information technology to mobile rounds, electronic medical records, all-in-one card payments, real-time in-hospital queries, radio frequency identification devices (RFID) barcode wristband identification, community monitoring, remote rehabilitation, and smart elderly care to explore the mouth [10]. However, how to integrate these scattered information technologies to more efficiently manage stroke patients throughout the entire process has yet to have clear guidance experience [11].

Regarding the typical research results of stroke robots, there is BLEEX (Berkeley Lower Extremity Exoskeleton) developed by the University of California, Berkeley [12] and the stroke robot HULC developed by Qi et al. [13] in conjunction with the University of California, Berkeley (Human Universal Load Carrier). Among them, the BLEEX robot has designed a back support, stroke mechanism, and power equipment to increase the soldier's walking ability and load capacity. At the same time, more than 40 sensors installed on the stroke complete the human-computer interaction of the control system. The HULC robot developed by Domingo [14] in conjunction with the University of California, Berkeley, adds an upper limb assisted stroke mechanism to the BLEEX robot to greatly improve the soldier's load capacity and combat capability. In addition, in Asia, Ahmadi et al. [15] of Nanyang Technological University (NTU) in Singapore have also developed a stroke robot for lower limb walking. The robot uses a hybrid control system, including power supply equipment, driving equipment, measurement systems, computers, wireless networks, and other equipment. At the same time, it collects the joint angles of the inner lower limbs while walking and provides assistance through the principles of physiological feedback and feedforward. In addition, many universities and research institutes around the world have carried out many researches on lower limb stroke robots for medical rehabilitation. A typical example is the “Lokomat” stroke rehabilitation robot developed by Sundmaeker et al. [16] at the Federal University of Technology Zurich (ETH) in Switzerland. Not only can it improve the treatment efficiency of acute ischemic stroke, it can also use telemedicine to contact hospital experts, manage physiological variables, improve hospital transportation decisions, and promote emergency care for other nervous system emergencies. Its efficacy has been clinically proven and has attracted many follow-up related studies. Kang et al.'s research [17] shows that the robot is composed of a weight loss system, a stroke system, a power and control system, and other supporting equipment: under the control of a computer, a linear motor and a crank-slider mechanism drive the hip and knee joints in stroke. At the same time, the ankle joint is designed with a passive adaptation mechanism [18]. The weight loss device elastically connected to the stroke system provides continuous support for the patient. The treadmill system provides coordinated movement for the human gait movement; the system adjusts the step according to the needs of the patient. At the same time, the active force of the patient is measured by the force sensor to adjust the output torque to adapt to the training needs of the patient in different rehabilitation stages and physical conditions [19]. In addition, the length of the mechanism of each joint part of the robot is adjustable to meet the body shape requirements of different patients and increase the compatibility of the rehabilitation system [20]. After the Lokomat robot appeared, related function development was constantly updated. In addition, there are many other research results of stroke rehabilitation systems, including the “Lopes” lower limb gait rehabilitation stroke robot developed by the University of Twente in the Netherlands [21], the “ALEX” lower limb gait rehabilitation stroke robot developed by the University of Delaware [22], and the Motorica stroke rehabilitation robot in the United States [23]. During the rehabilitation process, the system puts the patient in a tilted state with adjustable angle (tilt angle range: 0°–90°). At the same time, the patient's lower limbs can be gait with small amplitude through the traction mechanism of the thigh and the spring pedal mechanism of the foot. They move training to reduce the complications of bed rest and speed up the rehabilitation of the lower limb motor system and nervous system [24]. This mechanism combines the standing up bed with gait training, which increases the comfort of patients and is suitable for the rehabilitation needs of critically ill patients [25]. However, limited by the scope of the organization's activities, the system can only be used for small stride lower limb training [26]. At the same time, the driving method of the system determines that it can only achieve a single stepping action, which is not suitable for the development and use of other gait training functions [27].

Based on the technical requirements of community rehabilitation and family rehabilitation, this paper designs a stroke rehabilitation robot system that combines a stroke rehabilitation robot and a remote rehabilitation information management system. It uses IoT technology and is based on design methodology to realize the automatic generation of optimized rehabilitation strategies. It summarized the current research results. First, this article analyzes the rehabilitation needs of the stroke robot rehabilitation system, based on the concept of the Internet of Things, clarifies the specific structure of the rehabilitation system, and sorts out and proposes a comprehensive stroke rehabilitation robot system plan to adapt to the smart medical care in the construction of smart cities. It also explained the functional modules and network structure of the system and formulated the standardized use process under different conditions. After completing the analysis of rehabilitation goals and the system structure, this article carried out the overall design of the system and introduced the specific research work of each module, including the design and software design of the network database information management module and the design of the RFID recognition function module. The article also presented design and software design, SMS reminder GSM function module design and software design, camera remote monitoring function realization, robot terminal control, and information management module and focused on the realization of human-computer interaction control. In addition, the characteristics of each module need to be described. On this basis, the data model of the information system is established, and the rehabilitation process specifications for different patient states are given according to the relevant functions of different rehabilitation robots. At the same time, according to the design methodology and knowledge base management, a design process for generating the optimal rehabilitation strategy is given. This article proposes a remote stroke diagnosis and treatment service model based on the wireless Internet of Things, making full use of the advantages of modern information technology to improve the level of stroke diagnosis and treatment and promote the development of telemedicine. In view of the increasing incidence of stroke in China and the implementation of early stroke identification being not optimistic, this study proposes the use of the Internet of Things and the use of multitarget data collection, multiterminal information interconnection and connection, cloud computing intelligent data processing, and remote home monitoring under remote home monitoring. Under the multifactor and sign information comprehensive evaluation of early stroke identification and alarm system, a health management model is established, that is, a health management model based on the Internet of Things and cloud computing for early identification and early warning of ischemic stroke, to solve the early identification of ischemic stroke difficult question.

## 2. Construction of the Elderly Stroke Prevention and Nursing Management Model under the Medical Internet of Things

### 2.1. Basic Theory of Internet of Things

The concept of the Internet of Things can be traced back to 1999 and was proposed by Kevin et al. The International Telecommunication Union (ITU) discussed the concept and characteristics of the “Internet of Things” in its November 2005 report, as well as the difficulties it will face in the future development process, and released relevant results. In order to achieve the purpose of interaction between people and things, people use devices such as wireless sensors, RFID, GPS, and other devices to connect real-life objects to the Internet, and this process is called the old *J* of the Internet of Things. The continuous improvement of the infrastructure has led to the rapid development of the core technologies of the Internet of Things, and they have been applied in all aspects of daily life. Since different application service providers have different monitoring goals, a huge amount of monitoring data to be processed is generated. If it cannot be processed in a timely and efficient manner, it will cause serious waste of bandwidth resources in the network transmission process. Since the working status of each node of the Internet of Things cannot be guaranteed to be stable, there is a serious problem of uncertainty in the data of the Internet of Things.

Suppose the recognition frame is West, assuming the set function [0, 1] (the power set in the middle is 2 things) satisfies 2 conditions: *n*(*O*) = 0 and ∑*n*(*M*)=1; then the function *n* is called basic credibility distribution. The overall architecture of stroke unit can be divided into four parts: terminal layer, network layer, platform layer, and application layer. When there are many VM C, the basic credibility distribution value of *A* is *rt*(*M*), where *rt*(*M*) represents not the total credibility value of *M*, but an allocated value of the basic credibility of *M*. Sum the assigned values of all the subsets in *M* and express them with the reliability function to obtain the total reliability of *M*. Suppose that it represents a recognition framework reliability set function *A*: 2 in [0, 1] must meet 3 conditions at the same time: *A*(*O*) = 0; *A*(multi) = 1; when enough *c*, there is

(1) $$\begin{array}{c} u\left[x,y\right]>\sum u\left(x\right)-\sum u\left(x*i,y*i\right). \end{array}$$

The reliability is analysed again with the plausibility function. Suppose *A*: 2 in [0, 1] is a reliability function in 2, if the function day and function *S* are both in 2 [0, 1], when there is more VMC, *H* (*M*) = *A* (*M*), *S*: 1 − *A* (*M*), call the function *H* as the suspected function of *A,*. *s* is the plausibility function of *A*. It can be seen that the degree of suspicion is day (*M*) and the degree of plausibility is *S* (*M*). Suppose that *A*, and *A*, two reliability functions, are in the same recognition framework, and the assigned values of basic reliability are *n*, respectively, for its coking element. If ∑*n*. (*B*.) and *n*: (*C* − *j*) < 1, then the function *n* defined by formula (2) is the basic credibility distribution. When *n* ≠ *O*,

(2) $$\begin{array}{c} y\left(n\right)=\frac{\sum n\left(b\right)*n\left(c\right)}{1-\sum n\left(b\right)*n\left(c\right)}. \end{array}$$

When multiple reliability functions are in the same framework, their corresponding basic credibility distributions are 7, respectively. Assume that VM C is small, and *M* ≠ *O*. There is a basic credibility distribution, denoted by *n*, and then,

(3) $$\begin{array}{c} u\left(m\right)=k\sum n\left(m\left(i\right)\right)*\sum n\left(m\left(j\right)\right),\\ k={\left[\sum n\left(m\left(i\right)\right)\Lambda n\left(m\left(j\right)\right)\right]}^{-1}. \end{array}$$

For the data fusion of IoT nodes, each node in the IoT is regarded as a proposition, and the result displayed by the sensor with the functions of identification, judgment, and processing is the evidence corresponding to the proposition. If you want to integrate the data of multiple nodes in the Internet of Things, measure the collected data and then establish the corresponding basic probability distribution function as a credibility indicator. Each function and corresponding frame is called an evidence body, so every sensor in the IoT node is an evidence body. When calculating the normalization constant *K*, the increase in the number of assumptions will cause the amount of calculation to increase explosively, and the Dempster synthesis rule makes DS evidence theory a good solution to the problems of multisensor data conflicts and inconsistent opinions from multiple experts. Using Dempster merging rules to combine each evidence body into a complete evidence body under the same framework, this is the essence of IoT node data fusion. It demonstrates a *D*-s data fusion method based on IoT nodes, where *M* = 1, 2,…, *n*. (*M*) is the basic credibility distribution of *i* nodes, *i* = 1, 2,…, *z*, and is the new basic credibility distribution combined by the Dempster synthesis rule.

In the data fusion of multiple nodes, the huge amount of data makes the traditional calculation method difficult to apply. Let it be the result of combining all the evidence, and 1～n are the *n* pieces of evidence. The calculation method of combining the two evidences is used to deduce. Here, *z* represents not the total reliability value of *c*, but an assigned value to the basic reliability of *c*. Sum the assigned values of all the subsets in *e* and express them with the reliability function to obtain the total reliability of *e*. The calculation of the combination of *n* evidences is shown in the Figure 1, where the left side is the traditional direct calculation and the right side is the calculation of the recursive combination of *n* evidence. Suppose there is more recognition space = {elbow1, elbow2,…, elbow-*n* }. It is a variety of hypotheses, the evidence set *E* = {E1, E2,…, E*n*}, the weight set corresponding to each evidence which is *W* = {W1, W2,…, W3}, and conflict of each evidence *k*. According to the D-s evidence theory, the probability of conflict is defined as

(4) $$\begin{array}{c} z=\left(\sum c\left(i,j\right)-\sum e\left(i,j\right)\right)/\left(\sum c\left(i,j\right)+\sum e\left(i,j\right)\right),\\ c\left(i,j\right)=\sum n\left(i\right)*m\left(s\right)+n\left(j\right)*m\left(t\right),\\ e\left(i,j\right)=\sum n\left(j\right)*m\left(s\right)-n\left(i\right)*m\left(t\right). \end{array}$$

At this time, the original node weight is introduced, and the total weight form *W* = *m* × *k* − *o* × min is determined according to the size of the conflict probability. Among them, *W* − *i* is the smallest value among the original weights. The total weight here takes into account the conflict situation. Adjusted according to the total weight, the original weight minus the average of the total weight, that is, the weight of each piece of evidence minus the weight of the conflict part, is

(5) $$\begin{array}{c} v=c\left(i,j\right)*e\left(i,j\right)*z,\\ v\left(i,j\right)=\frac{v\left(i\right)*v\left(j\right)}{{\sum \left(v\left(i\right)*v\left(j\right)\right)}^{T}}. \end{array}$$

### 2.2. Medical Prevention and Nursing Management System Algorithm

Internet of Things data fusion algorithm is a technology for fusion processing of multisource data, which is the scope of intelligent information processing technology. By fully analyzing and integrating the data of each node, the best consistent estimate of the monitored object is obtained, which is more accurate and comprehensive than a single data source, so that users can make the right choice. After years of development of data fusion algorithms, some algorithms have formed more mature methods, and some algorithms are hotspots of scholars' research. Common data fusion methods mainly include classical probabilistic inference, Bayesian method, neural network, fuzzy set theory, and DS evidence theory.

(1) Classical probabilistic reasoning: the scope of classical probability discussion is limited to the case III1 of equal possible outcomes produced by random trials. Each test has a limited number of results, and the probability of the results is consistent. (2) Bayesian method: the Bayesian (Bayes) method was developed relatively early; the method is based on the maximum posterior and likelihood ratio test; if the prior probability can be calculated, Bayesian method will be a good solution. *A* is the result of combining all the pieces of evidence, and 1～n are the *n* pieces of evidence. The calculation method of combining two pieces of evidence is used to calculate the combination of *n* pieces of evidence. (3) Neural network: in recent years, the technology of neural network (neural networks) for data fusion has made great progress. The working principle of the neural network is similar to that of the human brain, simulating the thinking of the human brain. Different from the traditional set, each element in the fuzzy set has a corresponding membership degree. The degree of membership refers to the degree of certainty (or uncertainty) that an element belongs to this set. Therefore, the fuzzy set is described by the membership mapping function. The algorithm has the characteristics of simple parallel distributed computing, parallel distributed processing (fast speed), high fault tolerance, and data robustness. The neural network allows the input of multiple signals and the output of multiple variables. After system training, the data is allocated to the correct classification for output, which is suitable for multivariable systems. The neural network can input new data that has not appeared before and recognize it during the training process, so the algorithm can learn and adapt. The DS (Dempster Sharer) evidence theory is promoted on the basis of Bayesian method, introducing the concept of trust function and using multiple evidences. The specific algorithm flow chart is shown in Figure 1.

The steps of the *S* evidence theory method are Input—the target to be fused *M*, the trust function *n* − *i* (elbow) of *n* nodes, and the corresponding node weight training—and Output—the result of the fusion target. The steps are the following:

1. Calculate the conflict probability of each piece of evidence *n* − 1(*M*). Adjust the corresponding basic probability distribution according to the conflict probability, and get a new basic probability distribution.
2. Calculate *n* − *M* and *n*, the conflict coefficient *K* of (*M*). When *K* ≠ 1, call the D-s evidence fusion formula for data fusion to obtain the fusion data *n*(*C*).
3. Cycle *n* once or twice. Calculate the conflict coefficient *K* between *n*(*C*) and *n* − *m*(*M*). When *K* ≠ 1, call *D*. The evidence fusion formula updates the fusion data *n*(*C*).
4. The loop ends, and the final fusion result *n*(*C*) is obtained.

The entire software system is divided into five layers: the access layer, the resource scheduling layer, the data processing layer, the application support layer, and the application service layer. The vital signs remote transmission system is connected to a large amount of medical monitoring equipment through the network, and the patient's heart rate, respiration, and other physical signs data are collected through monitoring equipment such as electrocardiographs, ventilators, smart bracelets, and blood pressure monitors and transmitted back to the monitoring center through real-time network transmission. Real-time transmission of data is collected by medical equipment to the platform server, real-time diagnosis, and recording and saving of relevant data.  Figure 2 shows the specific model framework. We can span heterogeneous system architectures and network transmission protocols, seamlessly integrating the management applications of systems, networks, and services; the data processing layer is based on RMI (Java Remote Method Protocol) to implement data access services, which is convenient for program components to perform distributed computing; the application support layer uses Web Service to publish data subscriptions and gateway management services, with cross-platform and cross-language data interaction capabilities; the application service layer is implemented by using the Struts2 + Sprin93 + Hibernate3 framework, and the software system's hierarchical structure is divided into the domain object layer, data access object layer, business logic layer, controller layer, and presentation layer reducing the coupling between software codes and improving scalability.

The access layer is composed of the IoT gateway access server group, which is mainly responsible for processing the registration, login, data transmission, release, and other related requests of the IoT gateway, and can forward the data transmitted by the gateway to the corresponding data access server for further deal with. The access layer is only responsible for gateway access and data reception and forwarding and does not interact with the database. The number of gateways mounted on each gateway access server is dynamically balanced according to the performance of each server, the current load situation, and configuration parameters. A Hash algorithm is proposed to make the requests between the upper and lower layers consistent. The specific process: after the system web server receives the subscription request, then take the subscribed gateway ID to the corresponding data access server through the Hash algorithm. The elements between the frameworks flow with each other. The top layer is the server architecture, the middle layer is the module recognition and data sorting platform, and the bottom layer is the application terminal and feedback mechanism processing. We use the above high-quality algorithms to configure the number of data access servers in the configuration file to support the expansion of the number of servers. Each data access server keeps its own subscription list and does not require interaction. The subscribed request and the subscribed data are fixed on the same data access server, which can provide the query efficiency of system. A good Hash algorithm can ensure that the accessed gateway is evenly hashed on each data access server to achieve the effect of load balancing.

### 2.3. Optimization of the Stroke Protection Model under the Internet of Things

The users of the telemedicine system under the Internet of Things are divided into administrators, general users, and health experts. All three types of users need to pass identity authentication to use the system. Administrator user characteristics: manage the daily operation of the platform, manage the access of the IoT gateway, manage the registration, basic attribute entry, and authorization of the other two types of users, maintain and manage data, and be responsible for report generation. The remote stroke unit based on the wireless Internet of Things should meet the basic medical conditions of the stroke unit, and install cameras and microphones that can realize multiangle monitoring to facilitate the collection of video and audio information; we install wireless sensors to collect temperature, humidity, illuminance, and air quality for indoor environmental information.

The telemedicine system based on the Internet of Things is divided into three subsystems according to functions: the basic platform subsystem, the application platform subsystem, and the specific application subsystem. The application platform subsystem provides three major functions: user management, portal access, and application management. It is mainly responsible for managing users' usage rights, data access control, and classification display of user interfaces. At the same time, it provides users with personalized customization services for specific applications.  Figure 3 shows the distribution of various medical application services. The specific application subsystem provides specific medical-related services, including hypoxia analysis, arrhythmia analysis, electrocardiogram, blood pressure, blood pressure, blood oxygen, blood glucose, and fat and other medical applications, as well as online consulting function services.

The IoT gateway is generally deployed in residents' homes, in community health centers, or in mobile service vehicles. The IoT gateway access server can be deployed in each regional center, the dispatch server is accessed through the Internet or local area network and finally connected to the data access server, and the data collected by the gateway is forwarded to the data access server. The data access server, database server, and application server should be deployed in a local area network to ensure transmission speed and system operation efficiency. Application servers provide services to system users through the Internet. Combining business characteristics and needs, deploy various functional subsystems, database management software, gateway access software, data processing, and security authentication software in the business server as needed. The disk array mainly realizes the storage of system business application data and log backup data and is connected to the database server through a storage switch. The disk array performs redundant backup in the manner of RAID6 + hot spare disk to provide system security. In view of the high system requirements because of the stability and reliability of the database and application server, you can consider the use of dual-machine integrated data. Based on the Internet of Things telemedicine system design engineering master's degree thesis group design, the database server can be deployed in the form of dual servers and disk arrays. The database software adopts Oraclelog Enterprise Edition database service software, and the dual-machine cluster software chooses Oracle's high-availability real-time application cluster software (RAC).  Figure 4 shows the distribution of medical database values under the Internet of Things. They are deployed in various regional centers and access the dispatch server through the Internet or local area network and finally access data. We collect data separately through single-chip microcomputer and realize real-time data upload through NB-IOT module. When there is data to be sent, *M C U* sends in accordance with the priority and time sequence. When there is no data to send, the whole machine enters the standby state. The server forwards the data collected by the gateway to the system.

The database design process generally includes the following steps.

1. Demand analysis: fully understand the specific requirements of various potential users for data, operational requirements on business processes, and data integrity and security requirements.
2. Conceptual design: abstract entity data to define a comprehensive scheme and structure.
3. Logical structure design: design various tables of the database according to the entity model, and give the logical relationship between each other.

In response to the design requirements of the personal health monitoring platform, the system database design needs to comply with the following requirements:

1. Internet of Things related data: user's medical data, user's Internet of Things gateway information, Internet of Things gateway server, and other related information are stored in the information database of the Internet of Things data platform.
2. Application platform related data: user login information, application registration information, user application customization information, and first page board configuration information are all stored in the application platform information database.

## 3. Application and Analysis of the Elderly Stroke Prevention and Nursing Management Model under the Medical Internet of Things

### 3.1. Simulation of Model Weight Parameters

For people who are over 40 years old, a stroke risk screening assessment is carried out based on the following 8 risk factors (1 point for each item): (1) history of hypertension (blood pressure ≥140/90 mm Hg (1 mm Hg = 0.133 kPa)) or taking antihypertensive drugs; (2) heart disease such as atrial fibrillation and/or valvular disease; (3) smoking; (4) dyslipidemia; (5) diabetes; (6) rarely doing physical activities; (7) obviously overweight or obese (body mass index ≥26 kg/m^2^).  Figure 5 shows the fitting curve of medical data weights under the Internet of Things.

Stroke patients enter the stroke path immediately after admission and start standardized treatment. The image data can be transmitted without loss to ensure the accuracy of remote diagnosis. Physicians of the two parties communicate in real time through video, which can basically achieve the effect of face-to-face communication. The dedicated optical fiber keeps all data confidential, which can protect the privacy of patients to the greatest extent. In addition, the remote consultation system has added a medical wireless microphone (model: IMI-B2()) and a multimodal input kit (desktop) (model: IMI-G1 (10 microphones + XCM-1 (J mouse)) designed by the company. The consultation process can realize the entire voice input, and the consultation records and medical records will be generated accordingly at the end of the consultation. The important category of stroke TAST classification n1 is cardiogenic stroke. Atrial fibrillation is an important risk of cardiogenic stroke factors, and long-term ECG monitoring is a routine item in the etiology of stroke patients. After the content is determined, the plug-in design is carried out, and the corresponding MCU encodes the data format of the IC card, so that the IC card swiping time of the portable card reader and the card ID can be uploaded to the telecommunications platform and application server. If atrial fibrillation is detected, it is of great significance to the formulation of treatment plans and secondary prevention strategies.

We provide free hand-held ECG monitors for all stroke patients enrolled in the group, and monitor 5 regularly every day.  Figure 6 shows the error distribution of stroke data signal. The specific operation process is as follows: the patient downloads the palm ECG APP with his mobile phone and uses his mobile phone number to register the APP account. The plug-in ECG device connects the device to the patient's mobile phone by plugging into the audio port of the mobile phone. After the ECG data, the expert will read the ECG in the background and issue a report. After the patient's bed physician registers on the palm ECG cloud platform, the patient can search for the physician on the mobile phone client and click to send the report to the designated physician. The results can be viewed on the physician's platform and the patient can be responded to through the platform. All recorded ECG data will be stored in the cloud and recalled at any time. This mode is simple and feasible. Repeated operations can further improve the detection rate of atrial fibrillation.

Second-level preventive follow-up: all 20 stroke patients enrolled in the group were entered into the follow-up list after discharge and entered the follow-up phase to ensure the implementation of the secondary prevention of discharged patients.  Figure 7 shows the digital signal spectrum of the patient's stroke. The blue solid line in the figure represents the detected noise signal, and the red dashed line represents the denoising signal obtained after algorithm optimization. In the department link module, patients can instantly consult department physicians' introductions and outpatient schedules and make online outpatient appointments. There are 4 subitems: medication reminder and follow-up reminder. Follow-up records are presented in the form of questionnaires that can be designed and modified by physicians, which mainly include height, weight, blood pressure, blood sugar, diet, smoking, drinking, medication status, and modified Rankin Scale (RS) scores.  Figure 8 shows the polarization distribution of the stroke signal scale score.

However, a large proportion of stroke patients are elderly patients and do not use WeChat. To solve this problem, we apply an automatic telephone interview system specially designed by HKUST Company, which can dial up to 8 numbers at the same time through the cloud. Use predesigned questions (total 3 to 5 minutes) to conduct intelligent voice conversations, which can follow up simple but important data such as height, weight, blood sugar, blood pressure, medication status, and patient's current symptoms.

### 3.2. Example Results and Analysis

This study adopted a single-center, retrospective research method and selected NSTEMI patients who met the enrollment criteria and did not meet the exclusion criteria.  Figure 9 shows the stacked distribution of stroke electrical signal data. The data of the left sample group in the figure is denser than the right group, the data after the algorithm optimization accounts for more, and the corresponding score value is more excellent. Since the selected subjects are all NSTEMI patients, there is no low-risk population in the final risk stratification.

The patients selected in this study are all people above the intermediate risk. Before and after the establishment of the stroke center regional collaborative treatment system, the gender, smoking, diabetes rate, and previous angina pectoris, myocardial infarction, PCI history, family history, and history of cardiac insufficiency have been considered. The differences were statistically significant (*P* < 0.05). Among them, the subgroup analysis of the age variable shows that the age in each subgroup of group *A* is significantly larger than that of group B, and the difference is statistically significant (A1 group 68.48 ± 14.025 compared to B1 group 63.43 ± 13.432, *P* < 0.001; A2 group 75.15 ± 9.88 compared with B2 group 71.26 ± 10.58, *P* < 0.001; A3 group 60.85 ± 13.33 compared with B3 group 56.20 ± 11.71, *P* < 0.05). The subgroup analysis of the incidence of abnormal blood lipid metabolism showed that the A1 group was significantly lower than the B1 group [14.3% (6/42) vs. 38.6% (56/145), *P* < 0.001], and the A3 group was significantly lower than the B3 group [32.3% (50/155), *P* < 0.001]. Compared with 8.91 (1.63～48.44)], there was no significant difference between the two groups (*P* > 0.05); the Sym-to-FMC time of group B3 was slightly longer than that of group A3 [5.73 (1.38～21.25) versus 5.53 (2.38～42.05)], but there was no statistically significant difference between the two groups (*P* > 0.05).  Figure 10 shows the analysis of the abnormal incidence of stroke.

Through 9 months of practice and improvement, we have initially established a single-disease stroke smart medical consortium platform in accordance with the abovementioned plan. A total of 40 stroke patients and patients with risk factors enrolled in the group have been awarded top three hospitals in the five hospitals, high-quality medical services, and standardized community follow-up care management throughout the entire process. It breaks the time and space constraints, improves the work efficiency of physicians and the quality of medical services, and realizes community resource sharing and hierarchical diagnosis and treatment. All 20 patients in the stroke group have reached the 1-month follow-up period, and 153 of them have reached the 9-day follow-up period. A total of 12 patients' 9-day RS scores were actually obtained by follow-up on the official account platform, and the effective follow-up rate was 78.43%; 68 patients returned to the hospital for follow-up one month after the onset. The relevant data has been statistically complete and valid for one month. The return visit rate was 34%; 63 patients returned to the hospital for follow-up 9 days after the onset.  Figure 11 shows the medical treatment of stroke patients under the Internet of Things. The relevant data were perfect. The effective return visit rate was 41.1 8% in 90 days. According to the evidence theory method proposed in this paper, the system obtains the final basic credibility distribution; then we judged the rationality of the proposition based on indicators such as credibility and plausibility and output the decision result; finally, it is synthesized according to the traditional DS evidence theory formula. Among the 20 patients in the high-risk group, 16 have been followed up every 3 months since enrollment and have been closely observed until now, and the follow-up data is complete.

(1) Baseline information include age, gender, history of smoking, history of diabetes, history of hypertension, history of abnormal lipid metabolism, family history of early-onset coronary heart disease, history of angina, history of stroke, history of myocardial infarction, history of PCI, history of cardiac insufficiency, history of renal insufficiency, number of diseased vessels (left main, single, double, and three), eGFR at FMC, and risk stratification (very high risk, high risk, intermediate risk). (2) Time node indicators include the time from onset (the appearance of symptoms) to the first medical contact (Sym-to-FMC) and the time from the entrance of the patient to the gate of the PCI hospital to the start of the radiography (D-to-CAG). The rate of compliance, the time from first medical contact to transfer (FMC-to-Transfer), the proportion of PCI treatment within the time limit specified in the guidelines, and the total proportion of PCI treatment are also included. (3) Recent (in-hospital) prognostic indicators are in-hospital mortality, in-hospital heart failure, malignant arrhythmia, renal replacement therapy, gastrointestinal bleeding, and ventricular aneurysm. (4) One-year prognostic indicators are reinfarction rate, readmission rate, and 1-year mortality rate. (5) Economic benefit indicators are per capita hospitalization days and per capita hospitalization expenses.

There are some changes in limb motor function and Glasgow Coma Scale (GCS) scores and activities of daily living in the two groups before and 2 months after nursing.  Figure 12 shows the motor function scores of stroke patients after treatment. The Meyer Motor Function Evaluation Scale evaluates the upper and lower extremity motor function before and after the patient's care, with a full score of 100 points, of which the upper extremity motor function total score is 66 points and the lower extremity motor function total score is 34 points. The higher the score is, the better the recovery of the motor function of the limbs is. The higher the GCS score is, the more awake the stroke patient is. It is normal living ability: the patient's ability of daily living is judged by Barthel index, involving dressing, going up and down stairs, eating, etc. We use DS evidence theory to fuses data and adjust the weight of nodes according to the size of node weights and the probability of conflicts between nodes. The full score is 100 points. The higher the score is, the better the normal living ability of the patient is. It is statistical analysis: SPSS 20.0 software is selected for data proofreading, measurement data is described by mutual spider, and *t*-test is performed; count data is described by the number of cases (%), and *r* test is performed. *P* < 0.05 indicates that the difference is statistically significant.

## 4. Conclusion

This article uses the platform under the Internet of Things to provide raw medical data, patient health files, Internet medical service projects, etc. and uses cloud computing, big data, Internet of Things, artificial intelligence, and other technologies to build a single disease based on a safe and reliable hybrid cloud. It is a new type of smart medical consortium platform for stroke. In the results, a diagram of the whole-process management model for stroke patients was drawn; a community-level diagnosis and treatment system with smart community early screening for stroke, multidisciplinary remote consultation, smart follow-up evaluation, and clinical teaching synchronization was established; three levels of resource sharing provide a reliable and complete database for scientific research. The conclusion is that, with the support of cloud computing, big data, and other technologies, a safe and reliable Internet-based stroke smart medical consortium platform that meets the needs of multidisciplinary medical education and research integration and meets the needs of patients and medical care as the center has been constructed. The fourth-generation mobile communication network (4G) with high speed, small delay, good antinoise performance, and antimultichannel interference capability provides better conditions for the construction of a remote stroke prevention network based on the wireless Internet of Things. Therefore, the remote stroke prevention and treatment network will more effectively improve the level of stroke prevention and treatment at the first, second, and third levels, reduce the incidence and mortality of stroke, and provide remote diagnosis, treatment, consultation, and consultation for the prevention and treatment of other more diseases. We establish an information feedback system to collect opinions and suggestions from both doctors and patients at each node in the remote stroke diagnosis and treatment network in a timely manner, timely discover problems and hidden dangers in the process of remote stroke diagnosis and treatment services, and seriously solve them, so as to promote the quality of stroke diagnosis and keep treatment improving. The Internet of Things provides reliable technical support for the rapid application and landing of mobile stroke units. Through the in-depth integration of mobile stroke units and 5G network capabilities, it provides more possibilities for the rapid development of stroke first aid.

## Figures and Tables

**Figure 1:** Flow chart of medical protection algorithm under the Internet of Things.

**Figure 2:** The framework of the elderly stroke prevention and nursing management model under the medical Internet of Things.

**Figure 3:** Distribution of various medical application services.

**Figure 4:** Distribution of medical database values under the Internet of Things.

**Figure 5:** Fitting curve of medical data weights under the Internet of Things.

**Figure 6:** Signal error distribution of stroke data.

**Figure 7:** Digital signal spectrum of patients with stroke.

**Figure 8:** Polarization distribution of stroke signal scale score.

**Figure 9:** Stacking distribution of stroke electrical signal data.

**Figure 10:** Analysis of abnormal incidence of stroke.

**Figure 11:** Medical treatment of stroke patients under the Internet of Things.

**Figure 12:** Motor function scores of stroke patients after treatment.

## Data Availability

Data sharing is not applicable to this article as no datasets were generated or analysed during the current study.
